# Joint Detection of Tap and CEA Based on Deep Learning Medical Image Segmentation: Risk Prediction of Thyroid Cancer

**DOI:** 10.1155/2021/5920035

**Published:** 2021-05-31

**Authors:** Shaolei Lang, Yinxia Xu, Liang Li, Bin Wang, Yang Yang, Yan Xue, Kexin Shi

**Affiliations:** ^1^Sanmenxia Central Hospital of Henan Province, Sanmenxia, Henan 472000, China; ^2^Shaanxi Provincial People's Hospital, Taiyuan, Shaanxi 710068, China

## Abstract

In recent years, the incidence of thyroid nodules has shown an increasing trend year by year and has become one of the important diseases that endanger human health. Ultrasound medical images based on deep learning are widely used in clinical diagnosis due to their cheapness, no radiation, and low cost. The use of image processing technology to accurately segment the nodule area provides important auxiliary information for the doctor's diagnosis, which is of great value for guiding clinical treatment. The purpose of this article is to explore the application value of combined detection of abnormal sugar-chain glycoprotein (TAP) and carcinoembryonic antigen (CEA) in the risk estimation of thyroid cancer in patients with thyroid nodules of type IV and above based on deep learning medical images. In this paper, ultrasound thyroid images are used as the research content, and the active contour level set method is used as the segmentation basis, and a segmentation algorithm for thyroid nodules is proposed. This paper takes ultrasound thyroid images as the research content, uses the active contour level set method as the basis of segmentation, and proposes an image segmentation algorithm Fast-SegNet based on deep learning, which extends the network model that was mainly used for thyroid medical image segmentation to more scenarios of the segmentation task. From January 2019 to October 2020, 400 patients with thyroid nodules of type IV and above were selected for physical examination and screening at the Health Management Center of our hospital, and they were diagnosed as thyroid cancer by pathological examination of thyroid nodules under B-ultrasound positioning. The detection rates of thyroid cancer in patients with thyroid nodules of type IV and above are compared; serum TAP and CEA levels are detected; PT-PCR is used to detect TTF-1, PTEN, and NIS expression; the detection, missed diagnosis, misdiagnosis rate, and diagnostic efficiency of the three detection methods are compared. This article uses the thyroid nodule region segmented based on deep learning medical images and compares experiments with CV model, LBF model, and DRLSE model. The experimental results show that the segmentation overlap rate of this method is as high as 98.4%, indicating that the algorithm proposed in this paper can more accurately extract the thyroid nodule area.

## 1. Introduction

Thyroid cancer is a malignant tumor that originates in the thyroid follicular epithelium or parathyroid epithelial cells and is the most common malignancy of the head and neck. It often manifests as a painless mass of the neck or nodule. The treatment and prognosis of benign and malignant thyroid nodules are completely different [1, 2]. In this study, TAP serum and CEA were used to detect thyroid nodules in patients with thyroid nodules of type IV and above, with the aim of investigating the risk assessment of thyroid cancer in patients with thyroid nodules of type IV and above. Detection of TAP and CEA application value is in [3]. The segmentation of medical thyroid ultrasound images based on deep learning can be accurately calculated, while more objectively reflecting some characteristics of nodules, avoiding excessive subjective judgments, and giving more reliable results. Therefore, the medical segmentation algorithm based on deep learning in the ultrasound diagnosis of thyroid nodules has very important significance in the use of thyroid sarcoidosis [4].

In the research on the application value of TAP and CEA combined detection based on deep learning medical image segmentation in the risk estimation of thyroid cancer in patients with thyroid nodules of type four and above, many scholars have studied it and achieved good results. For example, Mohammadi et al. pointed out in their study that the expression of PTEN protein is downregulated in thyroid cancer, indicating that PTEN protein is closely related to thyroid cancer [5]. Xia et al. pointed out in their study that CEA is highly expressed in thyroid cancer, indicating that there is a certain correlation between serum CEA and thyroid cancer [6]. Cesareo et al. use a combination of principal component analysis (PCA) and minimum variance SVM to achieve the classification of hyperthyroidism, hypothyroidism, and normal thyroid, but the classification of several typical diffuse thyroid diseases is still in a blank state. No researchers have designed corresponding features according to the characteristics of different diffuse thyroid diseases and designed appropriate methods for classification [7].

In this article, the use of TAP and CEA to detect patients with thyroid nodules of type IV or above may increase the detection rate of thyroid cancer, reduce the rate of misdiagnosis and misdiagnosis, and reduce the risk of cancer. In this study, the use of TAP + CEA for the detection of patients with thyroid nodules of type IV and above is discussed, and it was found that the sensitivity, specificity, and accuracy of TAP + CEA detection are 96.84%, 96.79%, and 97.89%, which are higher than the sensitivity, specificity, and accuracy of serum TAP detection and serum CEA detection. The misdiagnosis rate and missed diagnosis rate of its combined test are lower than those of serum TAP test and serum CEA test, indicating that the use of TAP + CEA combined test to detect patients with thyroid nodules of type IV and above can improve the diagnostic efficiency of their thyroid cancer and reduce its missed diagnosis rate and misdiagnosis rate. The image segmentation grid model proposed in this document solves the problem of noise, initial contour sensitivity, and manual configuration of defined levels in the case of active edge contour segmentation. Experiments show that this shape is used to segment the nodules with ultrasound and can accurately separate the nodules; and, through some image segmentation evaluation parameters, segmentation accuracy is given objectively.

## 2. Based on Deep Learning Medical Image Segmentation, TAP and CEA Combined Detection Study on Thyroid Cancer Risk Prediction in Patients with Thyroid Nodules of Type IV and above

### 2.1. TAP and CEA Combined Detection Study on Thyroid Cancer Risk Prediction in Patients with Thyroid Nodules of Type IV and above

#### 2.1.1. Thyroid Nodules

The thyroid is a very important gland in vertebrates, and it is an endocrine organ. It is located below the thyroid cartilage in the neck of mammals and on both sides of the trachea. Thyroid cancer is the most common malignant tumor of the head, neck, and endocrine system. It is a differentiated thyroid cancer originating from the thyroid follicular epithelium. Thyroid nodule is a common thyroid disease, which is a mass that appears in the thyroid tissue after the abnormal proliferation of thyroid cells [8, 9]. Most thyroid nodules are not serious and do not cause abnormal symptoms. Thyroid nodules can be affected by people of all ages, and the incidence of women is higher than that of men. According to the severity of the thyroid gland, the thyroid gland can be divided into two categories, benign and malignant. Benign thyroid nodules are generally safer and can be observed and eradicated. Most of the malignant thyroid nodules are differentiated thyroid and require surgical treatment. According to clinical investigations, in recent years, the incidence of thyroid gland has increased rapidly worldwide, and the number of thyroid patients in my country is also increasing.

#### 2.1.2. TAP and CEA

TAP is an abnormal sugar-chain glycoprotein, also known as a tumor abnormal protein, which is mainly caused by new glycosylation caused by incomplete glycosylation or activation of new glycosyltransferases. It is a general term for glycoproteins and calcium-histone complexes emitted by tumor cells in the metabolic process. It is a metabolite of cancer cells. It is a common early screening method for tumors. When it reaches a certain level, it will discharge into the blood, and then the blood TAP is eliminated [10]. TAP is highly expressed in thyroid cancer and has certain diagnostic significance for the diagnosis and prognosis of precancerous condition. CEA is a carcinoembryonic antigen. It is metabolized by the gastrointestinal tract under normal conditions. When it enters the tumor state, the amount of carcinoembryonic antigen secreted by the tumor tissue will increase, and the carcinoembryonic antigen entering the blood and lymphatic circulation will also increase, passing through the blood and the secretion of tumor symptoms to detect carcinoembryonic antigen. The increase of its expression concentration can promote the abnormal proliferation and differentiation of follicular epithelium to increase the risk of metastasis of thyroid cancer cells. Studies have shown that TAP and CEA are closely related to thyroid nodules, and their detection can effectively judge the occurrence, development, and prognosis of various thyroid nodules and thyroid cancer. In this study, TAP combined with CEA was used to detect thyroid cancer patients with thyroid nodules of type IV and above. It was found that the levels of TAP and CEA in patients were elevated, indicating that the combination of the two can make a more accurate evaluation of thyroid classification. The prognosis of nodules has certain clinical significance.

#### 2.1.3. TTF-1

TTF-1 is thyroid transcription factor 1, which is normally expressed in thyroid follicular epithelial cells and bronchiolar epithelial cells. It is one of the members of the NKx-2 gene family that contains the homologous structure of internal transcription factors which has been researched in recent years. It can also be called NKX-2.1 or thyroid-specific enhancing binding protein. The positive expression of TTF-1 is a sign of hyperplasia and active function of thyroid tissue. PTEN protein can be expressed in a variety of tissues in early embryonic tissues. PTEN protein shows low expression in cancer tissues. The lack of expression may be closely related to the occurrence and development of tumors. As a glycoprotein, NIS is mainly located on the thyroid follicular epithelial cell membrane. NIS can use the energy produced by the “sodium-potassium pump,” which has the function of maintaining thyroid iodine uptake. The protein is also involved in the synthesis of thyroid hormone [11, 12]. NIS is not only expressed in the thyroid but also expressed in other parts of the human breast and prostate. Studies have shown that TTF-1, PTEN, and NIS are closely related to thyroid nodules and thyroid cancer, and their detection can more intuitively observe the occurrence and development of thyroid cancer and the classification of thyroid nodules. In this study, the protein expressions of TTF-1, PTEN, and NIS were detected and found that the amounts of TTF-1 and NIS proteins increased, and the amounts of PTEN proteins decreased, indicating that TTF-1, PTEN, and NIS proteins are closely related to thyroid nodules [13, 14].

### 2.2. Image Segmentation Algorithms and Models Based on Deep Learning

#### 2.2.1. Detailed Structure Analysis of Deep Neural Network

(1) *Sparse Convolution*. In a pure convolutional neural network, in which all convolution kernels are *k* × *k*, there is no pooling layer, and the receptive field of the unit corresponding to a convolution kernel is very easy to calculate. The size of the pixel block used to activate the cell is equal to *L* × (*K* − 1) + *K*, where *l* represents the layer number where this unit is located. The sparse convolution of signal *f* and kernel *k* with sparse coefficient *l* can be defined in the following form:

(1) $$\begin{array}{c} {\left(k_{l}^{*}f\right)}_{t}=\sum_{\gamma =-\infty }^{\infty }k_{\gamma }f_{t-l\gamma }. \end{array}$$

It can be seen that the difference from the traditional convolution is that the last subitem is changed from *f*_*t*−*γ*_ to *f*_*t*−*lγ*_, so that each convolution kernel is only combined with the elements at positions that are multiples of *l* in *f* contact.

(2) *Batch Standardization*. During the deep model training process, the parameters will need to be constantly updated with optimization algorithms such as backpropagation, and this update will inevitably cause changes in the distribution of input data at various levels. During the model training process, this change in the data distribution at the middle level of the network is commonly referred to as “Internal Covariate Shift.” In order to reduce this “internal variable transition,” it is usually necessary to set a small learning rate and carefully prepare the parameters.

Batch normalization is proposed to solve this problem. Specifically, normalization is performed in each dimension of each batch on the training set. The specific formula is as follows:

(2) $$\begin{array}{c} {\hat{x}}^{\left(k\right)}=\frac{x^{\left(k\right)}-E\left[x^{\left(k\right)}\right]}{\sqrt{\text{Var}\left[x^{\left(k\right)}\right]}}, \end{array}$$

where *x*=(*x*^(1)^ … *x*^(*d*)^), and the superscript indicates the dimension. Obviously this is a simple normalization similar to the whitening process. In order to avoid destroying the original distribution of the learned data, the learnable parameters *γ* and *β* are further introduced to transform and reconstruct the above formula:

(3) $$\begin{array}{c} y^{\left(k\right)}=\gamma^{\left(k\right)}{\hat{x}}^{\left(k\right)}+\beta^{\left(k\right)}. \end{array}$$

The forward propagation process of mini-batch standardization is as follows:

Input: the input value *x* of a batch: *B*={*x*_1…*m*_}, the parameters *γ* and *β* to be learned.
Output: {*y*_*i*_=*BN*_*γ*,*β*_(*x*_*i*_)}.
 process:
 Calculate the batch mean:
  (4) $$\begin{array}{c} \mu B=\frac{1}{m}\sum_{i=1}^{m}x_{i}. \end{array}$$
 Calculate the batch variance:
  (5) $$\begin{array}{c} \sigma_{B}^{2}=\frac{1}{m}\sum_{i=1}^{m}{\left(x_{i}-\mu B\right)}^{2}. \end{array}$$
 Normalized:
  (6) $$\begin{array}{c} {\hat{x}}_{i}=\frac{x_{i}-\mu B}{\sqrt{\sigma_{B}^{2}+\varepsilon }}. \end{array}$$
 Transformation reconstruction:
  (7) $$\begin{array}{c} y_{i}=\gamma {\hat{x}}_{i}+\beta \equiv BN_{\gamma ,\beta }\left(x_{i}\right). \end{array}$$

#### 2.2.2. Ultrasound Thyroid Nodule Level Set Segmentation Model Based on Deep Learning

(1) *The Model in This Article Model*. Through theoretical analysis and experimental verification, it can be clearly recognized that the global CV model cannot accurately segment the nodule images with complex backgrounds and blurred boundaries. Based on this, this paper proposes a model for the segmentation of learning score sets. This model adds a global directional energy element to the LBF model, which exceeds the sensitivity of the LBF model in the original contour and improves the segmentation of the fuzzy image boundary model [15, 16].

(2) *CV Model Based on Global Fitting*. The model uses the feature description method (grayscale, texture, etc.) of the image area information and adds these features to the active contour level set functional to drive the contour line closer to the image boundary. Compared with the traditional edge detection method, the region-based level set does not depend on the gradient information of the image (i.e., the edge detection operator) and overcomes the fuzzy boundary of the image or the edge leakage caused by the discrete image boundary to a certain extent. In addition, the level set based on regional information considers the image as the external and internal as a whole, so the CV level set model based on regional information is more sensitive to the initial contour.

(3) *Based on the Local Fitting LBF Model Method*. The universal mounting element in the CV model becomes the local mounting element, which significantly improves the ability to segment the blurred image with the border [17, 18]. However, the local customizer uses the local image information tightly and is not related to the global image. Therefore, the model depends more on the initial contour and is easy to fall to a local minimum during the evolution process, resulting in excessive segmentation and poor segmentation of the target boundary.

(4) *DRLSE Model*. Because the boundary of the ultrasound image is blurred and the weak boundary is often the contour of the target area, the accuracy of the active contour model based on the area is still not high in segmentation. Therefore, boundary-based active contours are gradually applied to image segmentation, and the most typical boundary model is the geodesic (GAC) model method. Although this method can be used to segment medical images, it is more complicated in numerical implementation and requires constant reinitialization, which is time-consuming [19, 20]. The model is further improved in the traditional penalty term function, so that the penalty term diffusion rate tends to infinity, the diffusion rate is a bounded constant, and the level set segmentation accuracy is higher.

## 3. Experimental Study of TAP and CEA Combined Detection Based on Deep Learning Medical Image Segmentation in Thyroid Cancer Risk Estimation in Patients with Thyroid Nodules of Type IV and above

### 3.1. Materials

400 patients with thyroid nodules of type IV and above were selected and screened by the Health Management Center of our hospital from January 2019 to October 2020 and diagnosed by puncture of thyroid nodules under B-ultrasound positioning and pathological examination for thyroid cancer. According to the test, 100 cases were divided into normal group, CEA positive group, TAP positive group, and CEA + TAP positive group. The normal group included 59 females and 41 males, aged from 29 to 87 years, with an average of (58.0 ± 23.2) years. The CEA positive group included 63 females and 37 males, aged 28 to 78 years, with an average of (53.0 ± 20.3) years; the TAP positive group included 51 females and 49 males with an age of 38 to 69 years, with an average of (53.5 ± 12.4) years; the CEA + TAP positive group included 46 females and 54 males, aged from 38 to 76 years, with an average of (57.3 ± 14.9) years. The general information of all patients is comparable.

Inclusion criteria are as follows: all patients who were diagnosed with thyroid cancer after puncture of thyroid nodules under B-ultrasound positioning and pathological examination.

Exclusion criteria are as follows: patients with heart, liver, kidney, and other organs' insufficiency; patients during pregnancy; patients with high levels of glycosylated hemoglobin such as diabetes; and patients with poor compliance. All patients and their families were aware of this study and approved by the ethics committee of our hospital.

### 3.2. Method

#### 3.2.1. Detection Method

In the TAP detection method, for making specimens, take 2 ml of fasting venous blood from all subjects, drop them on two slides respectively, push out two blood slides of uniform thickness, and place them on a water platform to let them dry naturally. Transplant the dried blood slice into a constant temperature and humidity environment and let it stand for 10 minutes. Use a dropper to draw the upper layer and drop it vertically onto the blood slice. The diameter of the drip spot is about 10 mm. The original “spots” are formed, where the reagents are dripped, which can be regarded as successful specimen preparation. For specimen detection, use an integrated reader microscope, with 4x ordinary achromatic objective lens, observe the three spots under the specimen on the display screen, look for specific forms of aggregates in the spots, use the TAP detection graphic system to take pictures of the particles, and use the software area to measure the particle size and record it.

In the CEA detection method, extract 2 ml of fasting venous blood from all subjects, centrifuge for 10 min, separate the serum after centrifugation, store it at −80°C for testing, use a fully automatic electrochemiluminescence instrument for electrochemical immunoassay, and strictly follow the instrument manual to avoid errors.

In the TAP + CEA detection method, the two detection methods are the same as above, and the statistics are combined after the two detections.

#### 3.2.2. Detection of TTF-1, PTEN, and NIS Expressions

Use PT-PCR to detect the expressions of TTF-1, PTEN, and NIS: extract total cell RNA, detect RNA purity and content, obtain cDNA after reverse transcription, use Primer 5.0 software to design primers, and use 2−▲▲Ct method for calculation. Set reverse transcription reaction conditions: 25°C for 10 min, 40°C for 60 min, and 85°C for 5 min; set amplification conditions: 94°C for 20 s, 72°C for 30 s, and 60°C for 30 s, 35 cycles, using 2−▲▲. The Ct method calculates the expression levels of TTF-1, PTEN, and NIS which need to be detected.

#### 3.2.3. Statistics of Inspection Results

Serum TAP, serum CEA, and serum TAP + CEA were checked for all subjects, the diagnosis, missed, and misdiagnosis status after the check were counted, and the missed diagnosis rate and misdiagnosis rate of the three inspection methods were compared.

#### 3.2.4. Diagnostic Efficiency

The following are statistics on the sensitivity, specificity, and accuracy of serum detection: Sensitivity = number of true positive cases/(number of true positive cases + number of false negative cases) × 100%. Specificity = number of true negative cases/(number of true negative cases + number of false positive cases) × 100%. Accuracy = (the number of true positive cases + the number of false positive cases)/total number of cases × 100%.

### 3.3. Experimental Research on Medical Images of Thyroid Nodules

In order to prove the rationality and effectiveness of the method proposed in this paper for ultrasonic thyroid nodule segmentation, this paper carried out different experimental analyses on the proposed model. The experiment is mainly divided into two parts: the first part verifies in detail the comparison of the segmentation results between the model in this article and the traditional DRLSE model. The second part compares the LBF model, CV model, DRLSE model, and the two methods proposed in this article. It shows that the method in this paper has a good effect on nodule segmentation. Finally, the segmentation accuracy of the two models in this paper is reflected by the calculation of segmentation accuracy.

### 3.4. Statistical Processing

SPSS 20.0 statistical software was used for analysis and processing. Measurement data are described by $\left(\bar{x}\pm s\right)$, LSD *t*-test is used for comparison between groups, *F* value test is used for comparison between multiple groups, percentage description is used for count data comparison, and chi-square test is used for comparison between groups. *P* < 0.05 is considered statistically significant.

## 4. TAP and CEA Joint Detection Based on Deep Learning Medical Image Segmentation in Thyroid Nodule Patients with Thyroid Cancer Risk Prediction Experimental Analysis of Type Four and above

### 4.1. Comparative Analysis of the Diagnosis Results of Deep Learning and High- and Low-Skilled Doctors

According to the test comparison results, the positive expected rate, negative expected rate, diagnostic sensitivity, diagnostic efficiency, and diagnostic specific indicators are calculated, respectively. These indicators are shown in Table 1.

It can be seen from Table 1 that the deep learning method surpasses the sonographer in all index comparisons. The positive expectation rate is 10.00% higher than that of senior sonographers, the negative expectation rate is 5.02% higher, and the diagnostic efficiency is 10.24% higher. The deep learning model constructed in this study is used to diagnose thyroid nodules more than sonographers and can assist physicians in real-time ultrasound diagnosis of thyroid examination.

This article makes a preliminary exploration of the application of deep learning technology in the field of ultrasound thyroid nodules. The results show that it is feasible to apply the deep learning method to the clinical auxiliary diagnosis of thyroid nodules in ultrasound images.

### 4.2. Detection of TAP and CEA Levels of Patients in Each Group

As shown in Table 2, compared with the normal group, the levels of TAP and CEA in the CEA-positive group increased (*P* < 0.05); compared with the CEA-positive group, the levels of TAP and CEA in the TAP-positive group increased (*P* < 0.05); and, compared with the TAP-positive group, the levels of TAP and CEA in the CEA + TAP-positive group increased (*P* < 0.05).

### 4.3. Detection of TTF-1, PTEN, and NIS Expressions

As shown in Table 3, compared with the normal group, the expressions of TTF-1 and NIS in the CEA-positive group increased, while the expression of PTEN decreased (*P* < 0.05). The expression of TTF-1 and NIS in tap positive group increased, but the expression of PTEN decreased (*P* < 0.05). Compared with the TAP-positive group, the expressions of TTF-1 and NIS in the CEA + TAP-positive group increased, and the expression of PTEN decreased (*P* < 0.05).

### 4.4. Comparison of the Detection Rates of Various Thyroid Nodules by Different Detection Methods

As shown in Table 4, TAP detected 352 cases of type IV thyroid nodules and 48 cases of type V thyroid nodules; CEA detected 352 cases of type IV thyroid nodules and 48 cases of type V thyroid nodules. There was no statistical difference between the detection methods of type IV and V thyroid nodules (*P* > 0.05); 389 cases of type IV thyroid nodules were detected by TAP + CEA, and 11 cases of type V thyroid nodules were detected. Compared with CEA test, it was statistically significant (*P* < 0.05).

### 4.5. Comparison of Missed Diagnosis and Misdiagnosis Rates by Three Detection Methods

As shown in Table 5, the missed diagnosis rate and misdiagnosis rate of serum TAP test were 11.25% and 5.75%, and those of serum CEA test was 11.75% and 6.25%. There was no statistical difference between the two (*P* > 0.05); compared with serum TAP and serum CEA detection methods, the missed diagnosis rate and misdiagnosis rate of serum TAP + CEA detection method decreased (*P* < 0.05).

### 4.6. Comparison of Sensitivity, Specificity, and Accuracy by Three Detection Methods

As shown in Table 6, the sensitivities of serum TAP detection and serum CEA detection were 85.25% and 89.85%, and the difference was not statistically significant (*P* > 0.05). The specificities of serum TAP detection and serum CEA detection were 85.06%, 88.00%. The accuracies of serum TAP detection and serum CEA detection were 86.28% and 87.61% (*P* > 0.05); compared with TAP detection and CEA detection, the sensitivity, specificity, and accuracy of TAP + CEA detection increased (*P* < 0.05).

The sensitivity, specificity, and accuracy of TAP + CEA are 96.84%, 96.79%, and 97.89%.

### 4.7. Experimental Comparison between the Traditional DRLSE Model and the Method in This Paper

This paper presents an image of a nodule with a low signal-to-noise ratio and a large background difference. At the right border of the nodule, there are some edges that are not distinguishable from the background. In the experiment, the binarized clustering threshold *T*_1_ = 0.9 in this paper, and the automatic level set evolution parameters are as follows: *λ* *=* 7.03 and Δ*t* = 0.3. The segmentation results of the method in this article are in good agreement with the segmentation of the experts. To be able to see the original outline of the cluster effect in binary format of this work, the original outline in dark red is shown in the image and the segmentation result is green. The original contour of the DRLSE model is located inside the nodule, which ensures that when the value of *α* is negative, the curve can be extended in only one direction. When repeated 60 times, the curve does not cross the line. However, in the final segmentation result, it can be clearly seen that the nodule boundary is exceeded in some places where the boundary is not clear. This is mainly because the boundary indicator function of the DRLSE model is not zero at some weak boundaries, which causes the curve to continue to expand forward, and finally the nodule boundary is not correctly segmented. The manual evolution parameters of the DRLSE model are *λ* = 9.2, Δ*t* = 4, and *a* = −0.5, and the experimental results are shown in Figure 1.

Figure 1(a) shows an experimental image with blurred borders. The contrast between the nodule and the background is more obvious, but, at the lower edge of the nodule, the distinction between the border and the background is not obvious. In the experiment, the binarized clustering threshold *T*_1_ = 0.54 in this paper, and the automatic level set evolution parameters are as follows: *λ* = 6.11 and Δ*t* = 0.9. Judging from the segmentation results, the difference between the second method in this paper and the expert segmentation results is relatively small. From the dark red initial clustering results of the image, it can be seen that the clustering results of the largest area in this paper are very close to the nodule boundary, so that the initial contour of the level set is more accurate than the initial contour manually set, which greatly reduces the number of evolutionary iterations of the level set in this paper. The initial contour of the DRLSE model is still set inside the nodule, the value of *a* is negative, and there is no boundary leakage when the iteration reaches 60 times, but, from the final evolution result, it can be clearly seen that there is oversegmentation at the lower boundary. There are two reasons for this: first, the DRLSE model is sensitive to noise; second, the function *g* that controls the curve at the boundary in the DRLSE functional is not zero at the weak boundary of the nodule.

### 4.8. Comparison Experiment of Segmentation Results and Segmentation Accuracy between Traditional Level Set and the Two Methods in This Article

The main reason is that there are both global segmentation items and local segmentation items in the model in this paper, and the sensitivity to the initial contour is greatly reduced. The segmentation results of the method in this paper are almost the same as the expert segmentation. It can be seen that the initial contour after clustering and binarization of the method in this paper is better than the initial contour manually set. The boundary stop function of the DRLSE model is better than the boundary stop function of the DRLSE model when segmenting weak boundaries. The experimental results are shown in Figure 2.

It can be clearly found from Figure 2 that the nodule area is not segmented in the upper right part. The experimental parameters are as follows: *λ*_1_ = 1.6, *λ*_2_ = 4.2, *v* = 0.04*∗*255*∗*255, *μ* *=* 1.4, and Δ*t* = 0.3. The boundary leakage of the DRLSE model also occurs when the boundary is blurred. The experimental parameters are as follows: *λ* = 7.2, *a* = 2.6, and Δ*t* = 1.1. From the experimental results, the two methods in this paper are relatively close to the expert segmentation results. Among them, the segmentation of the method proposed in this paper is different from the expert segmentation in some places, but the segmentation results of the method in this paper are different.

Table 7 shows the comparison between the number of iterations and the segmentation time when segmenting the three sets of images. From the data in the table, it can be seen that the model in this paper uses fewer iterations and the segmentation consumes less time.

It can be seen from Figure 3 that the number of iterations and time consumption of the method in this paper are longer than those of Method 1, which is mainly because the clustering part of the algorithm takes a certain amount of time. Overall, the two methods in this article are slightly better than other traditional level set algorithms. The following table shows the overlap rate data to further prove the accuracy of the experiment.

From the data in Figure 3, it can be clearly seen that the partition overlap rate of this method is as high as 98.4%, indicating the highest partition accuracy and the lowest error rate. The following conclusions can be drawn from the table: when looking for time efficiency, the method suggested in this article is the best choice for nodule segmentation, and when looking for accuracy, this method is the best choice.

## 5. Conclusion

This paper introduces FCM, SKFCM clustering algorithm, and DRLSE model algorithm. On this basis, a fusion segmentation algorithm using Fuzzy Kernel Clustering (SKFCM) and Improved Distance Regularization Level Set Model (DRLSE) is proposed. The model first uses a clustering method to roughly segment the nodule image and then selects the appropriate result type based on the clustering to binarize it and then uses the boundary of the binarized result as the initial contour of the level set, and the evolution parameters of the level set are calculated through the binarization region. The area calculates the evolution parameters of the level set, while improving the edge stop term of the traditional DRLSE model, replacing the penalty rule term of the traditional DRLSE model with Gaussian regularization, and applying it to ultrasonic thyroid nodule segmentation. The comparison between experiments and traditional level sets fully demonstrates the accuracy of the deep learning medical image segmentation algorithm proposed in this paper.

## Figures and Tables

**Figure 1:** Comparative experiment 1 between the DRLSE model and the method in this paper. (a) Original image. (b) Expert segmentation. (c) Method of this article.

**Figure 2:** Segmentation accuracy comparison (experiment 2). (a) Expert segmentation. (b) CV model segmentation. (c) LBF model segmentation.

**Figure 3:** Segmentation overlap rate (%).

**Table 1:** Comparison of diagnosis results between deep learning and high- and low-skilled doctors (%).

Object	Positive expectation rate	Negative expectation rate	Diagnosis sensitivity rate	Diagnostic efficiency	Diagnostic specificity
Sonographer (low)	73.42	80.62	98.32	73.25	19.04
Sonographer (high)	87.45	91.36	99.14	88.52	36.47
Machine learning	98.46	95.73	99.77	98.36	84.61

**Table 2:** Detection of TAP and CEA levels of patients in each group ($\bar{x}\pm s$).

Group	Number of cases	TAP	CEA
Normal group	100	89.02 ± 6.79	1.00 ± 0.23
CEA-positive group	100	103.03 ± 9.87^a^	2.54 ± 0.31^a^
TAP-positive group	100	138.56 ± 12.25^ab^	5.38 ± 0.51^ab^
CEA + TAP-positive group	100	210.01 ± 15.81^abc^	15.69 ± 4.01^abc^
*F*	—	68.591	55.261
*P*	—	0.001	0.001

Note: compared with the normal group, ^a^*P* < 0.05; compared with the CEA-positive group, ^b^*P* < 0.05; compared with the TAP-positive group, ^c^*P* < 0.05.

**Table 3:** Detection of TTF-1, PTEN, and NIS expressions in each group of patients $\left(\bar{x}\pm s\right)$.

Group	TTF-1	PTEN	NIS
Normal group	0.61 ± 0.02	1.69 ± 0.10	0.38 ± 0.05
CEA-positive group	1.02 ± 0.03^a^	0.97 ± 0.05^a^	0.81 ± 0.61^a^
TAP-positive group	1.23 ± 0.10^ab^	0.55 ± 0.02^ab^	1.46 ± 0.13^ab^
CEA + TAP-positive group	2.01 ± 0.14^abc^	0.29 ± 0.01^abc^	2.03 ± 0.20^abc^
*F*	56.310	78.252	75.216
*P*	0.001	0.001	0.001

Note: compared with the normal group, ^a^*P* < 0.05; compared with the CEA-positive group, ^b^*P* < 0.05; compared with the TAP-positive group, ^c^*P* < 0.05.

**Table 4:** Comparison of detection rates of various thyroid nodules by different detection methods (*n*, %).

Testing method	Type IV	Type V
TAP detection	352 (88.00)	48 (12.00)
CEA detection	341 (85.25)	59 (14.75)
TAP + CEA detection	389 (97.25)^ab^	11 (2.75)^ab^
*F*	35.161	39.568
*P*	0.001	0.001

Note: compared with TAP test, ^a^*P* < 0.05; compared with CEA test, ^b^*P* < 0.05.

**Table 5:** Comparison of missed and misdiagnosis rates by three detection methods (%).

Testing method	Missed diagnosis	Misdiagnosis
TAP detection	45 (11.25)	23 (5.75)
CEA detection	47 (11.75)	25 (6.25)
TAP + CEA detection	8 (2.00)^ab^	1 (0.25)^ab^
*F*	36.159	39.584
*P*	0.001	0.001

Note: compared with TAP test, ^a^*P* < 0.05; compared with CEA test, ^b^*P* < 0.05.

**Table 6:** Comparison of sensitivity, specificity, and accuracy by three detection methods (%).

Testing method	Sensitivity	Specificity	Accuracy
TAP detection	85.25	85.06	86.28
CEA detection	89.85	88.00	87.61
TAP + CEA detection	96.84^ab^	96.79^ab^	97.89^ab^
*F*	56.235	34.589	46.599
*P*	0.001	0.001	0.001

Note: compared with TAP test, ^a^*P* < 0.05; compared with CEA test, ^b^*P* < 0.05.

**Table 7:** Comparison of iteration times and segmentation times for three sets of images.

	—	Figure 1	Figure 2
Method of this article	Frequency	45	230
	Time consumption (s)	3.05	11.52

CV model	Frequency	320	440
	Time consumption (s)	6.43	16.53

LBF model	Frequency	220	610
	Time consumption (s)	5.70	16.73

DRLSE model	Frequency	160	270
	Time consumption (s)	4.04	12.64

## Data Availability

Data cannot be shared without permission from the data provider.
